# Conservation tillage improves productivity of sunflower (*Helianthus annuus* L.) under reduced irrigation on sandy loam soil

**DOI:** 10.1371/journal.pone.0260673

**Published:** 2021-12-21

**Authors:** Ahmad Sher, Muhammad Yasir Arfat, Sami Ul-Allah, Abdul Sattar, Muhammad Ijaz, Abdul Manaf, Abdul Qayyum, Ali Tan Kee Zuan, Omaima Nasif, Kristina Gasparovic

**Affiliations:** 1 College of Agriculture, Bahauddin Zakariya University, Bahadur Sub-Campus Layyah, Layyah, Pakistan; 2 Department of Agronomy, PMAS- Arid Agriculture University Rawalpindi, Rawalpindi, Pakistan; 3 Department of Agronomy, The University of Haripur, Haripur, Pakistan; 4 Department of Land Management, Faculty of Agriculture, University Putra Malaysia, Selangor, Malaysia; 5 Department of Physiology, College of Medicine and King Khalid University Hospital, King Saud University, Medical City, Riyadh, Saudi Arabia; 6 Institute of Plant and Environmental Sciences, Slovak University of Agriculture, Nitra, Slovakia; Harran Üniversitesi: Harran Universitesi, TURKEY

## Abstract

Sunflower production is significantly lower in arid and semi-arid regions due to various crop management problem. Conservation of tillage provides the most excellent opportunity to reduce degradation of soil reserves and increase soil productivity. The main objective of this study was to investigate the combined effects of conservation tillage and drought stress on growth and productivity of different sunflower hybrids. Experimental treatments included two sunflower hybrids (‘NK-Senji’ and ‘S-278’), two drought stress treatments (i.e., well-watered and drought stress at flowering and grain filling stages) and three tillage practices (i.e., conservation, minimum and deep tillage). The results indicated that morphological and physiological parameters, and yield-related traits were significantly (*P≤0*.*05*) affected by all individual factors; however, their interactive effects were non-significant. Among sunflower hybrids, ‘NK-Senji’ performed better for morphological, physiological, and yield-related traits than ‘S-278’. Similarly, conservation tillage observed better traits compared to the rest of the tillage practices included in the study. Nonetheless, conservation tillage improved growth and yield-related traits of hybrid ‘NK-Senji’ under drought stress. Hence, it is concluded that conservation tillage can improve the productivity of sunflower under low moisture availability. Therefore, conservation tillage could be suggested in the areas of lower water ability to improve sunflower production. Nonetheless, sunflower hybrids or varieties need thorough testing for their adaptability to conservation tillage and low moisture availability before making recommendations.

## Introduction

Sunflower (*Helianthus annuus* L.) is an annual oilseed crop cultivated in the world on 24.77 million hectares with a production of 44.31 million metric tons, which shares 8% of the world’s oilseed market [1]. Its achene consists of 40–50% oil and 17–20% protein; thus, have a clear ability to reduce the difference between production and consumption of edible oil. Sunflower s moderately tolerant to heat and water deficiency [2]; thus, has adaptability potential to semi-arid and subtropical regions of the world. Advances in development of sunflower hybrids in the recent years have dominated the open pollinated varieties in the field. Sunflower is usually grown in a wide range of climatic conditions ranging from temperate to tropical and semi-arid regions. Erratic rainfall patterns due to climate change and water shortage are faced during sunflower growth period. Therefore, most of the sunflower hybrids are area and climate-specific; hence, perform differently in different areas [3, 4]. Due to the reason, it is necessary to evaluate the growth and yield performance different hybrids under specific climatic conditions to choose the best suited one for higher yield and productivity.

Sunflower is a tropical and subtropical crop, often cultivated in dry land on supplemental irrigation [5]. Although sunflower is relatively tolerant to heat and drought stresses, extreme water deficiency severely affects its reproductive growth, resulting in yield losses [6]. Drought stress drastically reduced head diameter, achene yield, achene oil content and oil yield in sunflower [7–10]. The highest sunflower yield can be acquired by irrigating the crop at all critical growth stages, i.e., flowering and achene formation [10, 11]. Sufficient availability of water at early growth stages contributes towards good vegetative growth. However, low water availability at flowering and grain filling phases significantly reduces yield due to high transpiration requirements [10, 11].

Conservation of tillage provides an excellent opportunity to reduce the degradation of soil reserves and increase soil productivity [12]. Conservation tillage has attracted increased attention in recent years due urgent needs for erosion control and water conservation in various geographic regions of the world. Soil and water conservation-oriented tillage methods include conservation tillage, strip tillage, and mulch tillage [13]. Conservation tillage is an extreme type of tillage resulting in a negligible soil interruption [14, 15]. Conservation tillage is widely used in large-scale farming systems, where machinery is necessary for cultivation. Sustainable agriculture and increasing fuel costs in soil tillage inspire farmers to switch cultivation practices and urge them to find alternative tillage methods that are cost effective. The benefits of conservation tillage include enhanced surface water deposits, enhanced soil organic matter content, fertilizer recovery and protection from water and wind erosion [15–17].

Sunflower is a high yielding oil crop and serious efforts are required to increase its domestic production in Pakistan. This study was conducted to assess the productivity of sunflower hybrids sown under various tillage practices and water availability regimes. Major objective of study was to identify the most suitable tillage practice for better performance of sunflower hybrids under low water availability. The results would help to improve sunflower productivity under arid and semi-arid regions.

## Materials and methods

### Experimental site

A two-year (2018–19) filed study was carried out at experimental farm of Bahauddin Zakariya University, Bahadur Sub-Campus Layyah-Pakistan (30°57’N; 70°56’E; 151 m a.s.l). The region is subtropical semi-arid with cool winters and hot summers. The soil of the experimental site was sandy-loam having EC (154–156 dS m^-1^), pH (7.9–8.0), organic matter (0.67–0.69%), available phosphorus (9–10 ppm) and nitrate-nitrogen (1.6–1.8 mg kg^-1^). Average maximum and minimum temperatures, and mean rainfall during the growth period of sunflower in both years are given in Fig 1.

**Fig 1:** Average maximum and minimum temperature and rainfall during sunflower growth period during 2018 and 2019.

### Experimental treatments

The treatments comprised of two water availability regimes (i.e., well-watered and drought stress at flowering and grain filling stage), two sunflower hybrids (‘NK-Senji’ and ‘S-278’) and three tillage methods (i.e., conservation, minimum and deep tillage). Experiment was laid out according to randomized complete block design with split-split arrangement. Tillage practices, water availability regimes and sunflower hybrids were kept in main, sub and sub-sub plots, respectively. The net plot size was 3 m × 5 m. The crop was sown by hand drill without ploughing the soil in conservation tillage. The soil was ploughed with a cultivator to a depth of 10 cm and then crop was sown. Only the area where crop rows were sown was tilled, while the remaining field was not tilled. In deep tillage, whole experimental field was ploughed to 20 cm depth and then crop was sown.

### Cultivation practices

The crop was sown with hand drill by maintaining row-to-row distance of 75 cm. The crop was sown on March 8, 2018, and March 2, 2019. All agronomic practices were kept uniform following the local recommendations. Basal dose of N (90 kg ha^-1^) and P (60 kg ha^-1^) was applied at the time of sowing in the form of urea (46% N) and DAP (18% N, 46% P_2_O_5_) as source, respectively. The mature crop was harvested on May 2 and 7 during 2018 and 2019, respectively.

### Data collection

Randomly selected ten plants from each plot were measure for plant height from the base to the tip of plant and averaged. Stem diameter and head diameter were calculated with the help of Vernier Caliper.

Two central rows were harvested from each plot to count the number of achenes per head and biological yield. Harvested samples were sundried by keeping horizontal for few days. Dried samples were threshed and weighed to record achene yield in kg ha^**-1**^. Thousand-achene weight was counted by using the seed counter available in the Agronomy Lab.

Five plants were randomly selected from each plot were used to measure the chlorophyll index with the help of SPAD meter (CCM-200 plus). Fully developed leaves were used to measure physiological parameters (i.e., photosynthetic rate, transpiration rate, CO_2_ concentration and stomatal conductance) with the help of IRGA (InfraRed Gas Analyzer).

### Statistical analysis

The collected data were tested for normality and homogeneity of variance, which indicated that data were normally distributed. Differences among yeas were tested by paired t test, which indicated significant differences among years. Therefore, data of both years were analyzed and interpreted, separately. Three-way analysis of variance (ANOVA) was used to infer the significance in the data. Means were compared by least significant difference test where ANOVA indicated significant differences. The analyses were performed on Statistix statistical software.

## Results

### Morphological and yield traits

Morphological and yield traits were significantly (P≤0.05) affected by tillage practices, water availability regimes and sunflower hybrids. All three-way interactions were non-significant with some exceptions (Table 1).

**Table 1:** Analysis of variance (ANOVA) of morphological and yield-related traits of sunflower hybrids as influenced by various tillage practices and water availability regimes.

Source	df	Mean square													
		plant height		Stem diameter		Head diameter		Number of achenes head^-1^		1000-achene weight		Biological yield		Achene yield	
		2018	2019	2018	2019	2018	2019	2018	2019	2018	2019	2018	2019	2018	2019
Replication	2	388.1	383.7	1.31	1.01	4.0	3.6	111.1	8154	55.8	2043.5	644136	668344	359	3658
Tillage (T)	2	4148.6**	4131.4**	10.9**	20.52**	42.3**	36.7**	18065.6**	408076**	1680.6**	3164.8**	2113269**	1790519**	199905**	716325**
Main plot error	4	100.5	101.9	0.8	3.36	0.8	1.2	702.9	5905	98.2	8.7	164990	93303	2006	22517
Drought (D)	1	2085.4*	2070.3**	2.6**	19.05**	21.1*	8.8ns	12806.7**	340472**	1921.4**	1521.0**	1716100**	1964669**	1583822**	336593**
T × D	2	142.2 ns	144.3ns	0.8**	3.45ns	0.5ns	0.2ns	1751ns	4591ns	131.4ns	156.3ns	47308ns	46919ns	11482 ns	3930ns
Sub plot error	6	245.1	245.3	0.04	0.81	1.8	3.6	763.6	3776	63.6	63.7	95922	117061	2997	32957
Hybrids (H)	1	1089.0**	1100.0**	6.2**	20.69**	15.3**	43.6**	9900.2**	322056**	294.7**	940.4**	3336711**	3553225**	31506**	280017**
T × H	2	96.6ns	94.1ns	2.6**	3.57ns	4.6**	3.7ns	228.6ns	6265ns	7.2ns	10.1ns	46936ns	85908ns	505ns	75ns
D × H	1	40.1ns	38.0ns	0.5ns	0.02ns	3.3*	0.2ns	3154.7ns	42367**	283.4**	18.8ns	15211ns	145669ns	462ns	182ns
T × D × H	2	10.2ns	10.1ns	0.1ns	0.11ns	1.2ns	0.1ns	266.4ns	516ns	30.5ns	14.8ns	51586ns	54253ns	432ns	1339ns
Error	12	111.0	111.6	0.2	1.09	0.5	1.2	1052.4	4021	33.8	30.42	156453	173994	915	25937

Ns = non–significant;

* = significant at *P* ≤ 0.05;

**, *P* ≤ 0.01.

Conservation tillage significantly improved plant height (32.7 vs 31.4%), stem diameter (68.2 vs 78.2%), head diameter (62.2 vs 57.1%), number of achenes head^-1^ (6.7 vs 32.4%), 1000- achene weight (33.8 vs 42.7%), biological (12.8 vs 10.9%) and achene yield (18.8 vs 35.6%) compared to deep tillage system. Likewise, irrigation regimes significantly altered morphological and yield-related traits. Increase in plant height (12.4 vs 11.9%), stem diameter (54.5 vs 86.9%), head diameter (22.3 vs 13.3%), number of achenes head^-1^ (3.3 vs 16.4%), 1000 achene weight (20.8 vs 15.1%), biological (6.5 vs 6.4%) and achene yield (32.3 vs 13.7%) were observed under well-watered conditions compared to drought stress. Among sunflower hybrids, ‘NK-Senji’ performed better for plant height, stem/head diameter, number of achenes head^-1^, 1000 achene weight, biological and achene yield as compared to ‘S-278’ during both years (Table 2).

**Table 2:** The impact of different tillage practices and water availability regimes on morphological and yield-related related traits of sunflower hybrid type in 2018 and 2019.

Tillage Practices	Plant height (cm)		Stem diameter (cm)		Head diameter (cm)		Number of seeds head^-1^		1000-achene weight (g)		Yield (g ha^-1^)			
											Biological		Achene	
	2018	2019	2018	2019	2018	2019	2018	2019	2018	2019	2018	2019	2018	2019
**Conservation**	149.6 a	154.6 a	2.22 a	3.67 a	9.65 a	9.49 a	1225.7 a	1484.3 a	91.7 a	107.17 a	7391.7 a	7866.7 a	1623.8 a	1852.9 a
**Minimum**	127.3 b	132.2b	1.83 b	2.51 b	7.26 b	7.85 b	1182.3 b	1244.9 b	80.1 b	96.83 b	6959.2 b	7488.3 a	1481.4 b	1573.1 b
**Deep**	112.7 c	117.7 c	1.32 c	2.06 c	5.95 c	6.04c	1148.3 c	1121.7 c	68.0 c	75.33 c	6552.5 c	7094.2 b	1366.1 c	1366.1 c
***LSD (p ≤ 0*.*05)***	11.4	11.4	1.02	2.07	1.01	1.22	30.05	87.09	11.23	3.35	460.4	346.23	50.7	170.09
**Water availability regimes**														
**Well-watered**	137.4 a	142.4 a	1.53 a	3.14 a	8.39 a	8.28 a	1204.3 a	1380.9 a	87.2 a	99.61 a	7186.1 a	7716.7a	1694.2 a	1705.1 a
**Water stress**	122.2 b	127.3 b	0.99 b	1.68 b	6.86 b	7.29 b	1166.6 b	1186.4 b	72.6 b	86.61 b	6749.4 b	7249.4 b	1280.7 b	1500.7 b
***LSD (p ≤ 0*.*05)***	12.7	12.8	0.16	0.73	1.08	1.55	22.53	50.12	6.50	6.51	252.6	279.06	44.7	148.07
**Sunflower hybrids**														
**NK-Sinji**	135.3 a	140.4 a	1.67 a	3.17 a	8.27 a	8.88 a	1202.0 a	1378.2 a	82.8 a	98.22 a	7272.2 a	7797.2 a	1520 a	1685.6 a
**S-278**	124.3 b	129.3 b	0.84 b	1.65 b	6.97 b	6.68 b	1168.8 b	1189.1 b	77.0 b	88.0	6663.3 b	7168.9 b	1460.8 b	1509.2 b
***LSD (p ≤ 0*.*05)***	7.65	7.67	0.33	0.75	0.52	0.78	23.56	46.05	4.22	4.00	287.3	302.95	21.9	116.97

Letter sharing same number in each column does not have significant (P≤0.05) difference.

### Physiological traits

Physiological traits were significantly (P≤0.05) affected by individual effects of tillage systems, water availability regimes and sunflower hybrids. The two- and three-way interactions were non-significant with some exceptions (Table 3).

**Table 3:** Analysis of variance (ANOVA) of chlorophyll index and physiological traits of sunflower hybrids as influenced by various tillage practices and water regimes.

Source	df	Mean square									
		Chlorophyll content		CO_2_ concentration		Transpiration rate		Stomatal conductance		Photosynthetic rate	
		2018	2019	2018	2019	2018	2019	2018	2019	2018	2019
Replication	2	12.8	16.1	6445.4	6626.8	4.2	3.73	0.027	0.03	0.1	6.4
Tillage (T)	2	821.5**	832.2**	12970.4**	12904.4**	39.5**	37.7**	0.221*	0.22*	114.2**	99.3**
Main plot error	4	12.7	8.5	739.8	761.7	0.6	0.7	0.034	0.03	0.1	1.9
Drought (D)	1	99.3**	121.4**	17117.4**	17380.0**	18.2**	16.8**	0.036**	0.04**	49.5**	44.8**
T × D	2	10.4ns	10.8ns	1590.0ns	1577.0ns	0.3ns	0.4ns	0.021**	0.02**	1.2ns	0.7ns
Sub plot error	6	4.8	4.2	1141.9	1127.4	0.4	0.3	0.003	0.00	0.9	0.8
Hybrids (H)	1	220.0**	457.2**	17911.4**	17556.3**	34.1**	32.1**	0.134**	0.13**	63.3**	67.8**
T × H	2	14.2ns	11.0ns	3550.4**	3571.1**	0.4ns	0.5ns	0.102**	0.10**	0.4ns	1.8ns
D × H	1	11.8ns	5.2ns	2384.7ns	2352.3ns	0.1ns	0.3ns	0.004ns	0.004ns	0.1ns	0.1ns
T × D × H	2	11.3ns	9.9ns	392.7ns	399.1 ns	0.2ns	0.2ns	0.002ns	0.002ns	0.1ns	0.2ns
Error	12	19.4	15.9	614.6	636.6	1.1	1.0	0.004	0.004	0.4	0.9

Ns = non–significant;

* = significant at *P* ≤ 0.05;

**, *P* ≤ 0.01.

Among sunflower hybrids, ‘NK-Senji’ had higher photosynthetic rate, transpiration rate, CO_2_ quantity, and stomatal conductivity as compared to ‘S-278’. Likewise, under well water condition, better physiological traits were recorded compared to drought stress. Among tillage practices, conservation tillage system performed better as compared to other tillage during both years (Table 4).

**Table 4:** Chlorophyll contents and physiological attributes of two sunflower hybrids as affected by tillage practice and water availability regimes.

Tillage Practices	Chlorophyll index (SPAD values)		CO_2_ concentration		Transpiration rate		Stomatal conductance		Photosynthetic rate	
	2018	2019	2018	2019	2018	2019	2018	2019	2018	2019
**Conservation**	43.6 a	45.1 a	271.7 a	275.8 a	9.4 a	10.4 a	0.33 a	0.43 a	12.9 a	14.9 a
**Minimum**	34.1 b	37.4 b	239.3 b	243.5 b	7.6 b	8.6 b	0.09 b	0.19 b	9.7 b	11.8 b
**Deep**	27.1 c	28.5 c	205.9 c	210.3 c	5.8 c	6.9 c	0.08 b	0.18 b	6.8c	9.1 c
***LSD (p ≤ 0*.*05)***	4.03	3.31	30.82	31.28	0.90	0.94	0.20	0.20	0.43	1.55
**Water availability regimes**										
**Well-watered**	36.6 a	38.8 a	260.8 a	265.2 a	8.3 a	9.3 a	0.20 a	0.30 a	10.9 a	13.1 a
**Water stress**	33.2 b	35.2 b	217.2 b	221.2 b	6.9 b	7.9 b	0.14 b	0.23 b	8.7 b	10.8 b
***LSD (p ≤ 0*.*05)***	1.78	1.66	27.56	27.38	0.51	0.44	0.04	0.04	0.78	0.74
**Sunflower hybrids**										
**NK-Singi**	37.4 a	40.6 a	261.3 a	265.3 a	8.6 a	9.6 a	0.23 a	0.33 a	11.1 a	13.3 a
**S-278**	32.4 b	33.4 b	216.7 b	221.1 b	6.6 b	7.7 b	0.11 b	0.21 b	8.5 b	10.6 b
***LSD (p ≤ 0*.*05)***	3.20	2.89	18.00	18.32	0.74	0.72	0.04	0.04	0.43	0.69

Letter sharing same number in each column does not have significant (P≤0.05) difference.

## Discussion

Conservation tillage is any soil cultivation practice that leaves the crop resides (such as corn stalks or wheat stubble) in the fields prior to and after cultivation to mitigate soil erosion and runoff losses [13]. Conservation tillage systems may have been efficient than traditional tillage systems and result in improved soil quality. In current study photosynthetic rate, stomatal conductivity, carbon dioxide quantity, transpiration rate and chlorophyll pigments were higher under the conservation tillage compared to the rest of the tillage systems included in the study. Conservation tillage saves soil water, since the soil is relatively dense, with less water and soil nutrient leaching down [15–17], all of which contributed to better crop growth.

Better physiological growth resulted in improved morphological characteristics and yield (Table 3). Our results are in line with several previous findings [18, 19] regarding sunflower growth and yield under different tillage systems. Wang et al. [18] reported that conservation tillage confers stable microbial colonies and nutrient utilization which improve soil properties and results in improved growth and productivity of sunflower. Contrary to this, Paul et al. [15] recorded higher yield with maximum soil disturbance and minimum yield with zero tillage which attributed to the hard clay soil used in that experiment, while the soil in our experiment was sandy loam. Wasaya et al. [20] analyzed the effects of various tillage systems on soil properties in a four-year experiment and confirmed that different tilling practices did not alter soil bulk density, moisture content and hydraulic conductivity of sandy loam soils. In this analysis, therefore, better microbial activities and nutrient retention may result in higher productivity of sunflower under conservation tillage.

Drought is a physiological phenomenon that restricts water supply to fulfil its transpiration needs. Drought stress limits regular growth and reduces the morphological traits, such as stem dry weight (SDW), total dry matter (TDM), plant height, stem diameter [10, 19, 21, 22]. It suppresses stem elongation and eventually reduces the development of sunflower biomass. Decrease in biomass production under water deficit was noted in several studies on sunflower [10, 21, 22]. In our experiment, gas exchange parameters and chlorophyll content decreased under water stress conditions due to a reduced availability of water [10, 23] resulting in reduced plant growth and development. Water deficit compromised the formation of chlorophyll, photosynthesis, stomatal conductivity, and transpiration and resulted in declining plant biomass [22, 24]. Reduction in growth and development is accompanied by less carbon accumulation, unfair mineral nutrients, and abscisic acid (ABA) accumulation, which causes plant wilting [23, 24]. Reproductive stage is regarded as most drought sensitive stage of sunflower, and drought at this stage results in poor pollination and acene filling [25–28]. In the current study, under water deficiency, sunflower head diameter, achene yield, achene oil content and oil yield were significantly affected by the stress. Overall, drought stress affects all aspects of sunflower growth and development. In start, water deficiency stress decreases germination, stem elongation and leaf area [26, 27] and at reproductive stage, it results in pollen abortion resulting in empty acene [29–31].

## Conclusions

It is concluded that conservation tillage had positive impact on physiology and productivity of sunflower on sandy loam soil under normal and reduced irrigation. Conservation tillage seemed most economical option as it saves expenses incurred on tillage. Based on the results conservation tillage may be recommended for sandy loam soils of semi-arid regions for higher sunflower productivity. However, specific area and climatic conditions may also be considered for the recommendation of sunflower hybrids.
